The article "Association of body weight and physical activity with blood pressure in a rural population in the Dikgale village of Limpopo Province in South Africa" was retracted in 2013. Reasons: plagiarized data; no approval from the institution.

# Association of body weight and physical activity with blood pressure in a rural population in the Dikgale village of Limpopo Province in South Africa

**DOI:** 10.1186/1756-0500-5-118

**Published:** 2012-02-23

**Authors:** Seth S Mkhonto, Demetre Labadarios, Musawenkosi LH Mabaso

**Affiliations:** 1 Population Health, Health Systems and Innovation, Human Sciences Research Council, 134 Pretorius Street, Pretoria, 0002, South Africa; 2 Department of Medical Science, University of the Limpopo, Turfloop Campus, Fauna Park Polokwane, 0787, South Africa; 3 HIV/AIDS, STIs and TB, Human Sciences Research Council, 750 Francois Road, Durban, 4001, South Africa

## Abstract

**Background:**

Africa is faced with an increasing burden of hypertension attributed mainly to physical inactivity and obesity. Paucity of population based evidence in the African continent hinders the implementation effective preventive and control strategies. The aim of this study was to determine the association of body weight and physical activity with blood pressure in a rural black population in the Limpopo Province of South Africa.

**Methods:**

A convenient sample of 532 subjects (396 women and 136 men) between the ages 20-95 years participated in the study. Standard anthropometric measurements, blood pressure, and physical activity were recorded by trained field workers.

**Results:**

Anthropometric measurements showed that a high percentage of women were significantly (*p *< 0.001) overweight and obese than men. Hypertension was significantly high among women (38.1%) compared to men (27.9%). In the univariate analysis mean body mass index (BMI), waist circumference (WC), hip circumference (HC) and waist hip ratio (WHR) showed a significant positive association (*p *≤ 0.05) with systolic and diastolic BP in women, and only WHR was statistically significant in men. The odds of being hypertensive also increased with BMI, WC and WHR in both women and men, including HC in women. No relationship was found between physical activity and high blood pressure. In the multivariate analysis only increase in HC and WHR was consistently associated with increase in SBP in women and WHR with hypertension in men.

**Conclusions:**

The study findings indicate that women in this black South African rural population are overweight and obese than men and are at higher risk of hypertension as determined by selected anthropometric parameters.

## Background

High blood pressure (BP) or hypertension is a major public health problem worldwide, the disease is estimated to cause 7.1 million premature deaths globally [1]. Previously, the burden of disease was thought to be highest in developed countries. In fact, until recently, high blood pressure was thought to be rare in Africa. However, there is mounting evidence that developing countries are faced with an increasing burden of both hypertension and cardiovascular disease [2,3]. A number of studies have reported that hypertension is common in both rural and urban African populations due to lifestyle changes [4-7]. Hypertension has been associated with physical inactivity and obesity [8]. However, in most African countries including there is limited evidence base useful for designing and implementing effective preventive and control strategies [3]

In South Africa population based studies have also reported higher blood pressure among urbanized black Africans females compared to other race groups [9-12]. Even though there is an indication that the prevalence of hypertension is increasing in rural areas few studies have been conducted in these settings in the country [13]. In 1995 a demographic surveillance survey was established in the Digkale village in the Limpopo Province of South Africa and conducted one of the first measurements of physical activity and anthropometric parameters in a rural black population in the country [14]. Therefore the aim of this study was to investigate the association of body weight and physical activity with blood pressure using the Dikgale Demographic Surveillance System (DDSS).

The article "Association of body weight and physical activity with blood pressure in a rural population in the Dikgale village of Limpopo Province in South Africa" was retracted in 2013. Reasons: plagiarized data; no approval from the institution.

## Methods

### Study area

The Dikgale Demographic Surveillance System (DDSS) site is located in the Central Region in Mankweng district, about 40-50 km northeast of Polokwane, the capital city of Limpopo Province (Figure 1). All villages in Dikgale consist of communal grazing land some distance away from residential area. Settlements in Dikgale are a mixture of traditional mud huts, conventional brick houses and shacks with an estimated total population of 7900 people. Few households have water taps in the yards, but most of them fetch water from taps situated at strategic points in the villages. The area is impoverished with high unemployment and a large segment population working as migrant workers, farm labourers and domestic workers. The villages have poor infrastructure and most households have pit latrines with no organized waste disposal and roads are not tarred [14].

**Figure 1:** **Maps of South Africa and Limpopo showing the Dikgale District (shaded in black), the insert is the Dikgale Demographic Surveillence System site (shaded in blue) from Alberts et al**. [14].

### Study participants

Prior to field work Chiefs or Induna's in Dikgale were visited to explain the rationale behind the study and after the visit the Induna's informed the people in the villages. Initially, a random sample of 1000 subjects was generated from the DDSS relational database and distributed to trained fieldworkers. However, fieldworkers reported difficulty in contacting the subjects during house-to-house visits. Because of time and financial constraints, it was decided that fieldworkers would recruit participants house to house, at common meeting places, and through general mouth-to-mouth promotion of the survey. Therefore a total of 830 subjects were conveniently recruited between December 2005 and December 2007.

The article "Association of body weight and physical activity with blood pressure in a rural population in the Dikgale village of Limpopo Province in South Africa" was retracted in 2013. Reasons: plagiarized data; no approval from the institution.

Signed informed consent was obtained from all willing participants. Ethical approval was obtained from the Ethics Committee of the University of Limpopo (Turfloop Campus). Out of 830 participants we excluded 298 who were below 20 years of age and therefore, only 532 participants (396 women and 136 men) between 20 and 95 years of age were included in the analysis. Pregnant women or participants with renal disease were also excluded. Ten field workers were trained by research supervisor to take blood, measure physical activity and do anthropometric measurements in accordance with the standard procedures of the International Society for the Advancement of Kinanthropometry [15].

### Instruments and measurements

#### Anthropometry

All anthropometric measurements were taken twice and the average was recorded. Before the main survey, we conducted a small pilot study on 100 randomly selected students of different ages from the University of Limpopo to determine standard error of measurement and coefficients of variation between different observers. Once we were satisfied with the reliability of the measurements the main study began. Body weight was measured using an electronic scale (Fazzini, EB6371B, China) to the nearest 0.1 kg with the participants wearing light clothing and barefoot. Height was measured with the participants barefoot to the nearest 0.1 cm using a stadiometer and with their heads in the Frankfort plane. Body mass index (BMI) was calculated as weight divided by height squared (kg/m^2^). Waist circumference (WC) midway between the lower rib margin and the iliac crest was measured with the steel anthropometric tape to the nearest 0.1 cm extended around the waist parallel to the ground. The hip circumference (HC) was measured at the maximal circumference of the buttock with a steel tape to the nearest 0.1 cm. Circumferences were measured with the cross-hand technique, with the tape at right angles to the body and the readings were done on the right hand side. The waist to hip ratio (WHR) was calculated as WC divided by HC. Only one field worker in each village took the measurements to ensure uniformity and to avoid interstater variation.

The article "Association of body weight and physical activity with blood pressure in a rural population in the Dikgale village of Limpopo Province in South Africa" was retracted in 2013. Reasons: plagiarized data; no approval from the institution.

#### Physical activity

Physical activity was measured using a pedometer (New Lifestyles Inc., Kansas City, MO, USA) to calculate the average number of steps per day [16]. The device was mounted on the belt which the participants put around their waist on the right hand side except when bathing or sleeping. The participants were not visited or followed up they were instructed to wear the pedometer over nine consecutive days after which the data were downloaded.

#### Blood pressure

Blood pressure was monitored using the Omron electronic blood pressure equipment (Omron M5-I, R5-I and HEM-907) [17]. The blood pressure of the participants was measured three times with at least 2-3 min between successive measurements. All measurements were taken in a quiet room after the participants had been sitting in a chair for 5 min. Hypertension (high blood pressure) was defined as systolic (SBP) ≥ 140 mm Hg and diastolic blood pressure (DBP) ≥ 90 mm Hg [18].

### Statistical analysis

For statistical analysis the BMI (kg/m^2^) was classified into four categories: under-weight: < 18.5, normal weight: 18.5-24.9, over-weight: 25.0-29.9 and obese: ≥ 30.0 [12]. Physical activity measured by average step per day was categorized into five groups: sedentary: ≤ 5000, low active: 5000-7499, somewhat active: 7500-9999, active: 10000-12499 and very active: ≥ 12500 [19]. Descriptive statistics was used to define the characteristics of study participants. Differences between male and female participants were assessed using Wilcoxon-Mann-Whitney test for continuous variables and Chi-square test was used for categorical variables. Univariate linear regression analysis was used to assess the association of anthropometric parameters and physical activity to SBP and DBP. Binary logistic regression was used to assess the association of anthropometric parameters and physical activity to hypertension (normal or hypertensive) by estimating the odds ratio with 95% confidence interval (CI). Only variables significant in the univariate models for SBP, DBP and hypertension were fitted into multivariate models for each primary outcome. Variables were considered significant at a *p*-value ≤ 0.05. The analysis was done using STATA version 10 (STATA Corporation, College Station, Texas, USA).

## Results

### Characteristics of study participants

Anthropometric measurements showed that a high percentage of women were significantly (*p *< 0.001) overweight and obese compared to men. There was no statistically significant difference in SBP between women and men. However, women had significantly higher DBP than men. DBP among women varied between 48 and 157 mm Hg and between 55 and 115 mm Hg among men. Hypertension was significantly high among women (38.1%) compared to men (27.9). There was no significant difference in physical activity between women and men (Table 1).

The article "Association of body weight and physical activity with blood pressure in a rural population in the Dikgale village of Limpopo Province in South Africa" was retracted in 2013. Reasons: plagiarized data; no approval from the institution.

**Table 1:** Descriptive characteristics of female and male participants (n = 532)

Characteristics	Female (n = 396)	Male (n = 136)	All (n = 532)	
**Continuous variables**	Mean (SD)	Mean (SD)	Mean (SD)	*p*-value^±^
Age(years)	47.7 (18.7)	40.9 (19.2)	45.9 (19.0)	< 0.001
Height(cm)	158.9 (7.6)	167.8 (8.5)	161.2 (8.7)	< 0.001
Weight(cm)	68.6 (15.9)	64.9 (13.6)	67.6 (15.5)	< 0.018
Body mass index (kg/m^2^)	27.2 (6.2)	23.1 (4.8)	26.1 (6.1)	< 0.001
Waist circumference(cm)	86.4 (14.3)	77.6 (12.4)	84.2 (14.4)	< 0.001
Hip circumference (cm)	104 (14.3)	92.6 (11.2)	101.3 (14.5)	< 0.001
Waist-to-hip ratio	0.83 (0.08)	0.84(0.08)	0.83 (0.08)	0.330
Systolic blood pressure(mm Hg)	123 (24)	123 (20)	123 (23)	0.907
Diastolic blood pressure(mm Hg)	81 (14)	77 (11)	80 (13)	0.001
Physical activity (average steps/day)	11466 (5204)	12048 (4936)	11615 (5139)	0.173
**Categorical variables**	N (%)	N (%)	N (%)	
BMI categories (kg/m^2^)				
Underweight (< 18.5)	16 (4.0)	24 (17.7)	40 (7.5)	< 0.001
Normal weight (18.5-24.9)	148 (37.4)	75 (55.2)	223 (41.9)	
Overweight (25.0-29.9)	115 (29.0)	24 (17.7)	139 (26.1)	
Obese (≥ 30)	117 (29.6)	13 (9.6)	130 (24.4)	
Physical activity (average steps/day)				
Sedentary (< 4999)	40 (10.1)	13 (9.6)	53 (10.0)	0.205
Low active (5 000-7 499)	38 (9.6)	7 (5.2)	45 (8.5)	
Moderate active (7 500-9 999)	76 (25.0)	27 (19.7)	103 (19.4)	
Active (10 000-12 499)	99 (25.0)	32 (23.5)	131 (24.6)	
Very active (≥ 12 500)	143 (36.1)	57 (41.9)	200 (37.6)	
Hypertension (mm Hg)*				
Normotensive	249 (62.90)	98 (72.1)	347 (65.2)	0.053
Hypertensive	147 (37.1)	38 (27.9)	185 (34.8)	

Differences between women and men significant at *p *≤ 0.001, SD-Standard deviation, *systolic blood pressure ≥ 140 mm Hg and diastolic blood pressure ≥ 90 mm Hg

### Univariate analysis

Mean age showed a statistically significant positive association with SBP and DBP in both women and men (Tables 2 and 3). However, age was highly correlated with all other independent variables and was therefore excluded in subsequent analysis. Mean BMI showed a significant positive association with both SBP and DBP only in women, however, no significant association was found with BMI categories in both women and men. Both SBP and DBP were significantly and positively associated with WC, HC and WHR in women, and only WHR showed a significant positive association with both SBP and DBP in men. The association between categorical variables for physical activity (average steps per day) and blood pressure (SBP and DBP) were not plausible in both women and men. The risk of hypertension increased with BMI, WC and WHR in both women and men (Table 4). Increase in HC was only significantly associated with increased risk of hypertension in women. No statistically significant association was found between hypertension and categorical variables of BMI and physical activity in both women and men.

The article "Association of body weight and physical activity with blood pressure in a rural population in the Dikgale village of Limpopo Province in South Africa" was retracted in 2013. Reasons: plagiarized data; no approval from the institution.

**Table 2:** Univariate association of anthropometric parameters and physical activity with diastolic blood pressure (mm Hg) in women and men

Variables	Women (n = 396)				Men (n = 136)			
	
	*β*	95% CI		***p*-value**^**±**^	*β*	95% CI		***p*-value**^**±**^
Age (years)	0.654	0.546	0.763	0.000	0.354	0.186	0.522	0.001
Body mass index (kg/m^2^)	0.567	0.188	0.945	0.003	0.187	-0.530	0.905	0.606
Waist circumference (cm)	0.401	0.241	0.561	0.000	0.242	-0.032	0.515	0.082
Hip circumference (cm)	0.234	0.071	0.398	0.005	-0.039	-0.346	0.267	0.800
Waist-Hip-Ratio	70.121	40.898	99.344	0.000	59.885	21.145	98.625	0.003
Average steps/day	0.000	0.000	0.001	0.747	0.001	0.000	0.002	0.011
**BMI categories(kg/m^2^)**								
Underweight (< 18.5)	**	**	**	**	**	**	**	
Normal weight (18.5-24.9)	-17.590	-29.710	-5.469	0.005	0.127	-9.276	9.529	0.979
Overweight (25.0-29.9)	-13.230	-25.519	-0.941	0.035	1.375	-10.199	12.949	0.815
Obese (≥ 30)	-8.402	-20.679	3.874	0.179	1.756	-12.050	15.563	0.802
**Physical activity (average steps/day)**								
Sedentary (< 4999)	**	**	**	**	**	**	**	
Low active (5 000-7 499)	16.755	6.247	27.263	0.002	1.385	-17.241	20.010	0.883
Moderate active (7 500-9 999)	7.545	-1.517	16.606	0.102	2.570	-10.842	15.982	0.705
Active (10 000-12 499)	9.973	1.282	18.664	0.025	0.822	-12.245	13.889	0.901
Active (≥12 500)	8.349	0.052	16.646	0.049	7.771	-4.440	19.982	0.210

**First category taken as the reference group, *β *Regression coefficients, *CI *Confident interval, ^±^significant at ≤ 0.05

**Table 3:** Univariate association of anthropometric parameters and physical activity with systolic blood pressure (mm Hg) in women and men

Variables	Women (n = 396)				Men (n = 136)			
	
	*β*	95% CI		***p*-value**^**±**^	*B*	95% CI		***p*-value**^**±**^
Age (years)	0.263	0.195	0.331	0.000	0.190	0.095	0.284	0.001
Body mass index (kg/m^2^)	0.554	0.340	0.768	0.000	0.225	-0.176	0.626	0.269
Waist circumference (cm)	0.302	0.212	0.392	0.000	0.119	-0.035	0.272	0.128
Hip circumference (cm)	0.216	0.123	0.309	0.000	-0.073	-0.245	0.098	0.399
Waist-Hip-Ratio	40.122	23.222	57.022	0.000	40.538	19.173	61.902	0.000
Average steps/day	0.000	0.000	0.000	0.453	0.000	0.000	0.001	0.119
**BMI categories(kg/m^2^)**								
Underweight (< 18.5)	**	**	**	**	**	**	**	
Normal weight (18.5-24.9)	-9.667	-16.540	-2.795	0.006	-1.310	-6.539	3.919	0.621
Overweight (25.0-29.9)	-8.220	-15.188	-1.252	0.021	0.625	-5.812	7.062	0.848
Obese (≥ 30)	-1.145	-8.415	5.506	0.681	3.455	4.223	11.133	0.375
**Physical activity (average steps/day)**								
Sedentary (< 4999)	**	**	**	**	**	**	**	
Low active (5 000-7 499)	10.021	3.959	16.083	0.001	4.0.659	-5.733	15.052	0.377
Moderate active (7 500-9 999)	3.442	-1.785	8.670	0.196	1.083	-6.401	8.566	0.775
Active (10 000-12 499)	5.711	0.697	10.725	0.026	-2.269	-9.560	5.022	0.539
Active (≥ 12 500)	4.313	-0.473	9.100	0.077	2.652	-4.161	9.465	0.443

**First category taken as the reference group, *β *Regression coefficients, *CI *Confident interval, ^±^significant at ≤ 0.05

The article "Association of body weight and physical activity with blood pressure in a rural population in the Dikgale village of Limpopo Province in South Africa" was retracted in 2013. Reasons: plagiarized data; no approval from the institution.

**Table 4:** Univariate association of anthropometric parameters and physical activity with hypertension (mm Hg) between women and men

Variables	Women (n = 396)				Men (n = 136)			
	
	Odds Ratio	95% CI		***p*-value**^**±**^	Odds Ratio	95% CI		***p*-value**^**±**^
Age (years)	1.047	1.034	1.060	0.000	1.035	1.014	1.056	0.001
Body mass index (kg/m^2^)	1.048	1.013	1.084	0.006	1.092	1.010	1.181	0.026
Waist circumference (cm)	1.038	1.022	1.054	0.000	1.045	1.012	1.079	0.007
Hip circumference (cm)	1.020	1.005	1.035	0.009	1.018	0.984	1.054	0.296
Waist-Hip-Ratio	971.916	55.559	17002.150	0.000	2488.920	14.248	434771.3	0.003
Average steps/day	1.000	1.000	1.000	0.882	1.000	1.000	1.000	0.650
**Age Quartile categories(years)**								
**BMI categories(kg/m^2^)**								
Underweight (< 18.5)	**	**	**	**	**	**	**	
Normal weight (18.5-24.9)	0.480	0.170	1.356	0.166	0.500	0.180	1.387	0.183
Overweight (25.0-29.9)	0.456	0.158	1.310	0.145	0.824	0.242	2.797	0.756
Obese (≥ 30)	0.887	0.312	2.523	0.822	3.200	0.787	13.017	0.104
**Physical activity (average steps/day)**								
Sedentary (< 4999)	**	**	**	**	**	**	**	
Low active (5 000-7 499)	2.333	0.922	5.904	0.074	1.333	0.165	10.743	0.787
Moderate active (7 500-9 999)	0.891	0.384	2.069	0.788	1.667	0.365	7.607	0.510
Active (10 000-12 499)	1.517	0.690	3.333	0.300	0.933	0.200	4.347	0.930
Active (≥ 12 500)	1.502	0.706	3.196	0.291	1.417	0.346	5.800	0.628

**First category taken as the reference group, *CI *Confident interval

### Multivariate analysis

Categorical variables for BMI and physical activity were excluded due to lack of meaningful results in the univariate analysis. Only HC (*β *= 1.68, CI = 0.27-3.11, *p *= 0.020) and WHR (*β *= 252.70, CI = 69.06-436.34, *p *= 0.007) showed a significant positive association with SBP in women. The odds of being hypertensive increased significantly with WHR (OR = 597.04; CI = 0.97-0.36E06, *p *= 0.051) only in men. All the other selected variables showed no statistically significant association with SBP, DBP and hypertension in the final multivariate models.

The article "Association of body weight and physical activity with blood pressure in a rural population in the Dikgale village of Limpopo Province in South Africa" was retracted in 2013. Reasons: plagiarized data; no approval from the institution.

## Discussion

This study examined the association of anthropometric parameters, physical activity to blood pressure in women and men in a black South African rural population. Anthropometric measurements (BMI, WC, HC and WHR) showed that women were overweight and obese than men. While there was no difference in mean SBP between men and women, mean DBP differed significantly by sex and was higher in women (mean = 81 mm Hg) compared to men (mean = 77 mm Hg). Furthermore, hypertension was significantly high among women (38.1%) than men (27.9%). The 2002 South African Demographic Health Survey (SADHS) also found a had high prevalence of overweight and obesity among black women and this was associated with increased risk of hypertension [12-14].

In the current study univariate analysis identified central (BMI) and abdominal (BMI, WC, HC and WHR) measures of obesity as significant determinants of elevated SBP and DBP in women, and only WHR was significant in men. Hypertension also increased with increasing BMI, WC, and WHR in both women and men. HC showed a positive relationship with hypertension only in women. This is biologically plausible because in women most fat is distributed in the hips and in man around the waist [20]. However, no relationship was found between BMI categories and BP in both women and men. A study across three different populations in Africa found that although in general there was an increase in SBP and DBP with increasing BMI the risk of hypertension was not continuously distributed at all levels of BMI [21]. They found that there were BMI groups with an increased risk of hypertension and the cut of points varied markedly between men and women depending on ethnicity, biological, behavioural and environmental factors, including diet and nutrition, which have been implicated as determinants of high BP in different population groups [22,23].

Furthermore, in this study physical activity showed no clear association with blood pressure and hypertension. Marti et al. [24] and Manjoo et al. [25] also found no association between SBP and physical activity as measured by daily steps. Other studies in South Africa showed that average steps per day could not be used to define the intensity physical activity [26,27]. This can be attributed to the fact that physical activity levels are difficult to standardize and measure across populations in different countries [21,27,28].

In the final multivariate analysis only increase in HC and WHR was consistently associated with increase in SBP in women and WHR with hypertension in men. This is consistent with other studies which found WHR to be a strong independent indicator of hypertension than BMI for both sexes in some population groups [29-32]. It has been suggested that an increased WHR may reflect both a relative abundance of abdominal fat (increased WC) and a relative lack of gluteal muscle (decreased hip circumference) [33]. In addition, WHR not only shows body fat distribution but also reflects most of the lifestyle-related factors of an individual [34].

The article "Association of body weight and physical activity with blood pressure in a rural population in the Dikgale village of Limpopo Province in South Africa" was retracted in 2013. Reasons: plagiarized data; no approval from the institution.

The current study may be limited by potential risk factors or confounders which were not accounted for in the analysis such as dietary intake, substance abuse (alcohol and smoking) and other life style behavioural risk factors. The small sample size especially for men given the fact that the subsample of individuals used in the analysis was purposefully recruited makes generalization of the results difficult. Nevertheless, the findings of this study indicate that overweight and obese people especially women are more at risk of hypertension in this rural black population.

## Conclusion

Based on the finding of this study it is possible therefore as postulated by Grimm [35] that modernization of rural villages such as Dikgale has significantly changed lifestyle with consequent increase in obesity and hypertension. This highlights the importance of population based survey to monitor high blood pressure for effective prevention and control.

## Abbreviations

BMI: Body mass index; BP: Blood pressure; DBP: Diastolic blood pressure; DDSS: Dikgale Demographic Surveillance System; HC: Hip circumference; SBP: Systolic blood pressure; SADHS: South African Demographic Health Survey; WC: Waist circumference; WHR: Waist hip ratio.

## Competing interests

The authors declare that they have no competing interests.

## Authors' contributions

SSM was involved in data collection, performed initial data analysis and drafted the manuscript. MMLH assisted with statistical analysis, interpretation of data and revised the manuscript. DL made significant intellectual input, provided direction and helped revise the final manuscript. All authors read and approved the final manuscript.
